RETRACTED

# Mechanism of Dexmedetomidine Intervention on Neurogenic Inflammation in Cognitive Impairment Rats after Partial Hepatectomy

**DOI:** 10.1155/2022/8714221

**Published:** 2022-09-29

**Authors:** Zitan Zhang, Huiqun Jia

**Affiliations:** Department of Anesthesiology, The Fourth Hospital of Hebei Medical University, 12 Jiankang Road, Shijiazhuang, Hebei 050011, China

## Abstract

**Objective:**

To study the effect of dexmedetomidine on cognitive function in rats with cognitive impairment after partial hepatectomy and its mechanism.

**Methods:**

60 SD rats were randomly divided into 4 groups (*n* = 15): blank control group (CG group), sham operation group (Sham group), cognitive impairment model group (POCD group), and dexmedetomidine + cognitive impairment model group (DEX group). Rats in the POCD group underwent left lobe hepatectomy and intraperitoneal injection of the same amount of normal saline after resuscitation. Rats in the DEX group underwent left lobe hepatectomy and intraperitoneal injection of dexmedetomidine 50 *μ*g/kg. Group CG was not operated on and the same amount of normal saline was injected intraperitoneally. In the Sham group, liver resection was not allowed after the abdominal incision, and normal saline was injected intraperitoneally. Rats were injected every 24 hours for 5 consecutive days. Morris water maze (MWM) were used to evaluate the effects of dexmedetomidine on learning and memory ability of POCD rats. TUNEL method was used to detect apoptotic neurons in the hippocampus. INOS, Arg-1, IL-6, and TNF-*α*expression levels were detected. Western blot detects the expression level of TNF-*α*, Bcl-2, and NF-*κ*B protein.

**Result:**

Compared with the CG group, the escape latency of the other three groups was prolonged on the 5th day after the operation, and the number of crossing the platform was reduced. Compared with the Sham group, the escape latency of the POCD group and DEX group was significantly prolonged, and the number of crossing the platform was significantly reduced on day 5 (*P* < 0.05). Compared with the POCD group, the DEX group shortened the escape latency and increased the number of crossing the platform on the 5th day (*P* < 0.05). It shows that the spatial learning and memory function of rats has been restored to a certain extent.The number of iNOS and Arg-1 positive cells in the POCD group and DEX group was higher than that in the control group, and the number of Arg-1 positive cells in the DEX group was higher than that in the POCD group (*P* < 0.05). Western blot results the expression of Bcl-2 and NF-*κ*B protein in POCD group, and DEX group was higher than that of the sham group (*P* < 0.05). The expression of Bcl-2 and NF-*κ*B protein was the most in POCD group. The expression of Bcl-2 and NF-*κ*B protein in DEX group was lower than that in POCD group (*P* < 0.05).

RETRACTED

**Conclusion:**

Behavioral results showed that the learning and cognitive ability of POCD model rats after hepatectomy was impaired, and inflammatory factors and activated microglia were found in the hippocampus of POCD rats. Dexmedetomidine may improve the brain function of POCD rats by inhibiting neuronal apoptosis,partly through NF-*κ*B apoptosis pathway.

## 1. Introduction

Postoperative cognitive dysfunction (POCD) is a common postoperative complication in elderly patients undergoing general anesthesia. In this study, rats with cognitive impairment after partial hepatectomy were used as the research vehicle. After successful modeling, hippocampal region was used as the research object to understand the pathophysiological changes of hippocampal cells and tissues after cognitive impairment, and explore the expression characteristics of neurogenic inflammation and the activation of some classical apoptotic channels in this model. To study the effect of dexmedetomidine on the expression of inflammatory factors in the brain through the treatment of dexmedetomidine intervention. To investigate the effect of dexmedetomidine on the activation phenotype of microglia, and to explore the process of dexmedetomidine regulating the changes of different inflammatory states in the brain and regulating cognitive impairment, so as to provide more experimental basis for the mechanism of neurogenic inflammation of POCD and the safety of clinical anesthesia in aging patients.

Dexmedetomidine is a selective a2-adrenoceptor agonist. It hyperpolarizes noradrenergic and reduces norepinephrine release by activating pre- and post-synaptic a2-adrenoreceptors within the central nervous system, resulting in a sympatholytic effect. Dexmedetomidine administration produces sedation and anxiolysis, exerting its inhibitory effect on noradrenergic neurons in the locus coeruleus, and has minimal effects on respiratory drive. This study aimed to study the effect of dexmedetomidine intervention on neurogenic inflammation in cognitive impairment rats after partial hepatectomy.

## 2. Materials and Methods

### 2.1. Preparation of POCD Animal Model

Rats fasted for 12 hours before the operation. Rats were anesthetized with 1% pentobarbital sodium. After shaving the epidermal hair and disinfecting the surface of the abdominal skin, an incision about 1.5 cm long was made along the midline. The upper abdomen was opened to expose the liver, and the left hepatic duct and artery were ligated with 0 silk thread. The liver was partially resected before ischemia in the median and left lobes. The peritoneum and skin were sutured with silk threads, respectively. During the operation, arterial blood oxygen partial pressure (PO_2_) was maintained at 100~120 mmHg, and arterial blood carbon dioxide partial pressure was maintained at 35~45 mmHg. During the operation, the temperature of the rats was maintained at 37 °C, and 5 ml of sterile normal saline was injected into the abdominal cavity before closing the abdomen to compensate for the evaporation of body fluid, body fluid loss, and bleeding during the operation. The animals after surgery were placed in an incubator until resuscitation. Our study was approved by the institutional review board of the hospital and was conducted in accordance with the ethical principles originating from the Declaration of Helsinki.

RETRACTED

### 2.2. Animal Grouping and Treatment

Sixty 18-month-old SD rats (bred in the animal laboratory of Tianjin Nankai hospital) weighing 260-420 g, half male and half female, were randomly divided into four groups: (A) blank control group (CG group) (*n* = 15, intraperitoneal injection of the same dose of normal saline for 1-5 days); (B) sham operation group (Sham group) (*n* = 15, rats were anesthetized and abdominal incision was performed without hepatectomy, then the incision was sutured, and the same dose of normal saline was injected intraperitoneally 1-5 days after modeling); (C) cognitive impairment model group (POCD group) (*n* = 15, intraperitoneal injection of the same dose of normal saline 1-5 days after modeling); and (D) dexmedetomidine + cognitive impairment model group (DEX group) (*n* = 15, intraperitoneal injection of dexmedetomidine 50 (*μ*g/kg) per day 1-5 days after modeling.

### 2.3. Behavioral Experiments

Rats were first trained for 5 days. Morris water maze test was carried out 1, 3, and 5 days after the operation. The fourth quadrant was located in the experiment. In the place navigation test, Put the rat into the water, explore freely for 60 sec, and record the time when the rat successfully boarded the underwater hidden escape platform, which is recorded as the escape latency. Those who board the hidden platform within 60 seconds and stay for 10 seconds are deemed to have successfully boarded the platform; if the rats failed to board the platform successfully, they were guided to the platform and stayed for 10 sec. At this time, the escape latency was recorded as 60 sec. Each rat was trained four times a day, with an interval of no less than 60 min. The quadrant order of training was random and different. In the space exploration experiment, on day 5, remove the underwater platform in quadrant IV, put the rats into the pool with the same method from the midpoint of the opposite quadrant, and record the number of times the rats crossed the original hidden escape platform within 60 sec. The experiment was carried out from 8 : 00 to 14 : 00 every day, during which the rats were treated with heat preservation.

RETRACTED

### 2.4. Material Acquisition

One hour after the behavioral experiment, the rats were anesthetized by intraperitoneal injection of 2% lidocaine. After deep anesthesia, the rats were fixed on the operating table in a supine position, opened their chest, fully exposed their hearts, punctured into the ascending aorta at the left ventricular position, cut open the right atrial appendage, perfused with about 300 ml of normal saline at room temperature, rinsed from the left ascending aorta for about 15 minutes, and then perfused with about 300 ml of 4% paraformaldehyde (pH = 7.4) through the ascending aorta for cardiac lavage. The lavage speed was first fast, then slow, and finally fixed for 40-50 minutes. After the whole body of the rat was stiff, the rat was decapitated, and then the brain tissue was completely removed with surgical forceps. Compared with the stereotactic map of the rat brain, the coronal plane was cut at 1 and 6 mm after the optic chiasma, and the hippocampus of the rat brain was taken and trimmed to a size of about 1.0 ×. For the tissue block with a thickness of about 0.3 cm and a thickness of 1.0 cm, the trimmed tissue block is fixed in 4% paraformaldehyde fixation solution for 24 hours. Gradient absolute ethanol (50-100%) is used for gradient dehydration, and each gradient concentration of ethanol is dehydrated for 2 h. After dehydration, soak the tissue block in a xylene transparent agent for tissue transparency treatment. The transparent tissue block was immersed in paraffin two times, and the soaking time of each time was 3H. Put the tissue block completely soaked in wax into the embedded mold box for cooling and fixation. Use a slicer to cut the wax block in 4-6 *μ*M thick, perform continuous coronal slices, fish the slides with polylysine-treated slides, bake them in an oven at 50 °C, and store them at room temperature for standby.

### 2.5. HE Staining of Hippocampal Tissue Sections

Hippocampal tissue was stained with hematoxylin solution using a VS120 optical microscope 200 ×. Observe the staining results of the sections under the objective lens, and take photos. The morphological changes in cortex and hippocampus tissues and neurons were observed.

### 2.6. Detection of Apoptosis in the Hippocampus

After dewaxing and hydration of slices, use the TUNEL method, and operate in strict accordance with the instructions of the kit. DAPI counterstained the nucleus, the nucleus stained by API was blue in UV excitation, the Roche kit was labeled with FITC fluorescein, and the positive apoptotic nucleus was green.

RETRACTED

### 2.7. Detection of iNOS, Arg-1, IL-6 and TNF-*α* by Immunohistochemistry Expression

The brownish-yellow particles or stained brownish yellow that is expressed in the cytoplasm or nucleus of cells with complete structure, clear location, and clear staining contrast are judged as positive. Each slice was randomly selected to observe under high magnification (200×) of five mutually non-overlapping visual fields of the hippocampus, and the immunohistochemical positive cells were calculated. The intensity of the positive degree was semi-quantitatively analyzed by the image Proplus 6.0 digital medical image analysis system, and the results were shown by the integrated optical density (IOD/area) value (Table 1).

### 2.8. Western Blot Detection of Bcl-2, NF-*κ*B Protein Expression Level

Hippocampal tissue proteins were extracted from frontal and parietal lobe brain tissues 2 mm before and after optic chiasma. Automatic chemiluminescence analysis system (Tanon 5200, Shanghai) was used to detect the chemiluminescence of the target protein, the exposed bands were saved, and the gray value of the protein bands was analyzed by gel Pro analyzer software.

### 2.9. Statistical Analysis

Continuous normally distributed data are expressed as the means ± SDs.

All statistical calculations were carried out using SPSS statistical software.. *P* values < 0.05 were considered significant.

## 3. Result

### 3.1. The Results of Behavioral Experiment

The experimental results showed that compared with the CG group, the escape latency of the other three groups was prolonged on the 5th day after operation, and the number of crossing the platform was reduced. Compared with Sham group, the escape latency of POCD group and DEX group was significantly prolonged, and the number of crossing the platform was significantly reduced on the 5th day (*P* < 0.05), indicating that the modeling was successful. Compared with the POCD group, the DEX group shortened the escape latency and increased the number of crossing the platform on the 5th day (*P* < 0.05). It shows that the spatial learning and memory function of rats have been restored to a certain extent (Figures 1–3).

### 3.2. HE Staining Results

The brain tissue of the CG group is rich in the cerebral cortex, with a regular and dense arrangement, rich matrix, and uniform staining. The vessel cavity is normal, the vessel wall is smooth, the morphology of nerve cells is regular, and the structure has not changed significantly. There was no significant change in vascular morphology in the Sham group. In the POCD group, the shape of neuronal cells changed, the cytoplasmic staining decreased, the nuclei with deeper staining appeared, there was a clear gap between cells, and there were necrotic neuronal cells around. Compared with the cognitive impairment group, the DEX group had the same pathological changes, such as enlarged cell gap and neuronal cell necrosis, but the degree was significantly reduced, and the pathological damage to the cerebral cortex gradually weakened (Figure 4).

RETRACTED

### 3.3. DEX Significantly Decreased the Number of Positive Apoptotic Cells

In the POCD group, under the light microscope, the apoptotic cells can be seen in all parts of the hippocampus, the death-positive cells can also be seen around the injured area, and the positive apoptotic nucleus is green. In the DEX group, the number of positive cells decreased significantly. Under the microscope, only scattered apoptotic cells could be seen in the hippocampus of the sham group and CG group. According to the TUNEL rule, the number of apoptotic cells in the DEX group was less than that in the POCD group, and the statistical difference between groups was significant (*P* < 0.05) (Figure 5).

### 3.4. The iNOS and Arg-1 Positive Cells in the POCD and DEX Group Were Higher than Control Groups

Cells with brown or yellow staining are regarded as a positive expression. The number of IL-6 and TNF-*α* positive cells was the largest in the POCD group, and the inflammatory response was the strongest. The number of positive cells in the DEX group was lower than that in the cognitive impairment group. In the sham group, there was only a slight inflammatory reaction and positive cell process scattering. CG group can only see weak positive expression (Figures 6–9). The results of immunohistochemical detection of iNOS and Arg-1 showed that the number of iNOS and Arg-1 positive cells in the POCD group and DEX group was higher than that in the control group and the number of Arg-1 positive cells in the DEX group was higher than that in POCD group (*P* < 0.05) (Figures 10–13).

### 3.5. Bcl-2, NF-*κ*B in POCD Group and DEX Groups Were Higher

Western blot results the expression of Bcl-2 and NF-*κ*B protein in POCD group, and DEX group was higher than that of the sham group (*P* < 0.05). The expression of Bcl-2 and NF-*κ*B protein was the most in POCD group. The expression of Bcl-2 and NF-*κ*B protein in DEX group was lower than that in POCD group (*P* < 0.05) (Figures 14–16).

## 4. Discussion

Surgical trauma can cause the expression of inflammatory factors in the body to rise, such as IL-1, IL-6, and TNF-*α.* It is the most important cytokine that mediates inflammatory response. These inflammatory factors destroy the blood-brain barrier and cause the response of brain macrophages through the blood-brain barrier, thereby affecting the function of the brain [1]. The earliest inflammatory factor is TNF-*α*. It is also a key factor in a series of inflammatory reactions. In this experiment, the expression of inflammatory factors in different groups was studied. The highest expression levels of the inflammatory factors TNF-*α* and IL-1 were found in the POCD group. The expression of inflammatory factors decreased after dexmedetomidine intervention, which was consistent with the behavioral performance of experimental rats. The experimental results showed that compared with the CG group, the escape latency of the other three groups was prolonged after operation and the number of crossing the platform was reduced. Compared with Sham group, the escape latency of POCD group and DEX group was significantly prolonged, and the number of crossing the platform was significantly reduced. Compared with the POCD group, the DEX group shortened the escape latency and increased the number of crossing the platform. It shows that the spatial learning and memory function of rats have been restored to a certain extent. It is concluded that dexmedetomidine can reduce the inflammatory response of the central nervous system and reduce and improve the occurrence of postoperative central nervous system nerve injury.

RETRACTED

Microglia are innate immune cells of the central system. When the central nervous system receives external stimulation, microglia and astrocytes are passively activated [2]. Microglia can be divided into pro-inflammatory M1 type and anti-inflammatory M2 type according to their functions after being activated [3]. By TNF-*α*, the activation of microglia is called M1 macrophage [4], which is characterized by CD86, iNOS, CD16, and CD32. Another type of M2 macrophage, whose common characteristic phenotypes are CD204, CD206, CD16, Ym1 and arginase 1 (Arg-1). M1 macrophages mainly release proinflammatory factors and cytotoxic mediators, causing neuronal damage and further aggravation, resulting in the progressive death of neurons; M2 macrophages have neuroprotective effects such as inhibiting the inflammatory response and promoting tissue regeneration [5].

Through the data of this experiment, we observed that the expression of iNOS in the POCD group was the most, followed by the sham group, which was significantly higher than that in the blank control group. After dexmedetomidine intervention, the expression of iNOS decreased significantly, indicating that the release of inflammatory factors in the brain led to the activation of M1 microglia and the pathological process of cognitive impairment. The expression of Arg-1 in the DEX group was significantly higher than that in the POCD group, which confirmed the effect of the expression of two different subtypes of microglia on brain function. It shows that dexmedetomidine can promote the functional phenotype transformation of microglia and protect brain function.

RETRACTED

Some scholars have confirmed that dexmedetomidine can inhibit the activation of rat microglia and reduce the release of inflammatory mediators by inhibiting NF-*κ* B pathway in microglia. [6]. In the physiological resting state, NF-*κ* B and I *κ* B binding, is stable in the form of inactive dimer in the cytoplasm. When cells are stimulated, such as TNF- *α* Equifactorial action, I *κ* B kinase (IKK) is activated to promote I *κ* B phosphorylates [7] so that NF- *κ* B is activated, dissociated into p65 and P50 and transferred from cytoplasm to nucleus, participating in the transduction and transcription of a variety of cytokines [8]. NF-*κ*B has the recognition site of the iNOS mRNA promoter. After the cascade amplification of the signal pathway, the transcription level of the iNOS gene increases [9]. The activity of iNOS is enhanced, and finally, is generated. [10] A large amount of not accumulated in cells can cause DNA damage, leading to diaphragm mitochondrial dysfunction and contraction failure, and then affect the metabolism of neurons, leading to neuronal apoptosis. Bcl-2 is an important factor in cell apoptosis. In this experiment, the expression of Bcl-2 and NF-*κ*B protein was significantly higher in POCD group than that of other groups. The expression of Bcl-2 and NF-*κ*B protein decreased in DEX group but was still higher than that of the control group. Combined with the change of iNOS expression level, it shows that the stimulation of inflammatory factors increases neuronal apoptosis and affects brain function, while the effect of dexmedetomidine on inhibiting neuronal apoptosis and improving brain function may be through NF-*κ*B channel.

## 5. Conclusions

Behavioral results showed that the learning and cognitive ability of POCD model rats after hepatectomy was impaired and inflammatory factors and activated microglia were found in the hippocampus of POCD rats.

After dexmedetomidine intervention, it enhances the activation of microglia in the brain of normal aging rats, promotes the transformation of microglia functional phenotype, and participates in the regulation of the pathological process of neurogenic inflammation.

The release of inflammatory factors caused by neurogenic inflammatory lesions in the hippocampus activates NF- *κ* B apoptosis pathway of neuronal cells.

RETRACTED

Dexmedetomidine may improve the brain function of POCD rats by inhibiting neuronal apoptosis partly through NF-*κ*B apoptosis pathway.

## Figures and Tables

**Figure 1:** The moving track of rats in four groups on the 5th day in water maze spatial probe test.

**Figure 2:** The number of crossing the platform of rats in four groups in spatial probe test ($\overset{¯}{x}\pm s$) (*n* = 15).

**Figure 3:** Escape latency of rats in four groups in place navigation test ($\overset{¯}{x}\pm s$) (*n* = 15).

**Figure 4:** Representive HE staining of the hippocampus of CG/Sham/POCD/DEX rats (magnification, ×200).

**Figure 5:** Representative immunofluorescence images of apoptosis of hippocampal neurons of CG/Sham/POCD/DEX rats (magnification, x200). Green: TUNEL; blue: DAPI.

**Figure 6:** Representive immunohistochemical images of TNF-*α* positive cells in the hippocampus of CG/Sham/POCD/DEX rats at 200×magnification.

**Figure 7:** Expression of TNF-*α* positive cells in hippocampus of each group ($\overset{¯}{x}\pm s$) (*n* = 15).

**Figure 8:** Representive immunohistochemical images of IL-6 positive cells in the hippocampus of CG/Sham/POCD/DEX rats at 200×magnification.

**Figure 9:** Expression of IL-6 positive cells in hippocampus of each group ($\overset{¯}{x}\pm s$) (*n* = 15).

**Figure 10:** Representive immunohistochemical images of iNOS positive cells in the hippocampus of CG/Sham/POCD/DEX rats at 200×magnification.

**Figure 11:** Expression of iNOS positive cells in hippocampus of each group ($\overset{¯}{x}\pm s$) (*n* = 15).

**Figure 12:** Representive immunohistochemical images of Arg-1 positive cells in the hippocampus of CG/Sham/POCD/DEX rats at 200×magnification.

**Figure 13:** Expression of Arg-1 positive cells in hippocampus of each group ($\overset{¯}{x}\pm s$) (*n* = 15).

**Figure 14:** Expression of Bcl-2 and NF-*κ*B protein in the hippocampus in four groups.

**Figure 15:** Expression of Bcl-2 protein in the hippocampus in four groups ($\overset{¯}{x}\pm s$) (*n* = 15).

**Figure 16:** Expression of NF-*κ*B protein in the hippocampus in four groups ($\overset{¯}{x}\pm s$) (*n* = 15).

**Table 1:** Comparison of the expression of TNF-*α*, IL-6, iNOS, and Arg-1 positive cells in the hippocampus among four groups ($\overset{¯}{x}\pm s$) (*n* = 15).

	TNF-*α*	IL-6	iNos	Arg-1
CG	0.0242 ± 0.0198	0.0091 ± 0.0072	0.0016 ± 0.0006	0.0026 ± 0.0025
Sham	0.0159 ± 0.0085	0.0061 ± 0.0054	0.0074 ± 0.0018^a^	0.0023 ± 0.0013
POCD	0.0390 ± 0.0103^ab^	0.0204 ± 0.0118^ab^	0.0160 ± 0.0088^ab^	0.0022 ± 0.0069^ab^
DEX	0.0173 ± 0.0178^c^	0.0110 ± 0.0093^c^	0.0082 ± 0.0068^ac^	0.0115 ± 0.0105^c^

Note: Compared with group CG, ^a^*P* < 0.05; compared with group Sham, ^b^*P* < 0.05; and compared with group POCD, ^c^*P* < 0.05.

RETRACTED

## Data Availability

The data used to support this study is available from the corresponding author upon request.
